The article "The Correlation between Obstructive Sleep Apnea and Retinal Vein Obstruction: A Meta-Analysis and Systematic Review" was retracted in 2023. Reasons: signs of a paper mill; suspected computer-generated content; unreliable results or conclusions; concerns about the data.

# The Correlation between Obstructive Sleep Apnea and Retinal Vein Obstruction: A Meta-Analysis and Systematic Review

**DOI:** 10.1155/2022/8065629

**Published:** 2022-07-12

**Authors:** Ziwen Qin, Xiang Li, Hanyu Ren, Wei Song, Longlong Su, Xiaoling Gao

**Affiliations:** ^1^Second Clinical Medical College, Shanxi Medical University, Taiyuan 030001, China; ^2^Department of Respiratory and Critical Care Medicine, The Second Hospital of Shanxi Medical University, Taiyuan 030001, China

## Abstract

Despite of inadequate evidence, previous studies have demonstrated a potential correlation between obstructive sleep apnea (OSA) and retinal vein occlusion (RVO). In this study, a meta-analysis is conducted to investigate the correlation between OSA and RVO. Databases are searched for relevant literatures up to July 14, 2021, including PubMed, Embase, Cochrane, Web of Science, CNKI, WanFang, VIP, and Chinese Biomedical Literature Database (CBM). The odds ratio (OR) and 95% confidence interval (CI) are estimated to evaluate the correlation between OSA and RVO. Six articles were finally enrolled, including 36,086 subjects from 5 case-controlled studies and 1 cohort study. It is clearly evident that the RVO risk is higher among OSA patients than non-OSA patients (OR = 3.24, 95% CI = 3.24). The results of sensitivity analysis indicate that the present meta-analysis is robust and reliable. Furthermore, Egger's test for publication bias is performed with *P* = 0.195, and the results reveal no significant publication bias. The findings demonstrate that OSA is significantly correlated with RVO, and OSA is a risk factor for RVO.

## 1. Introduction

Obstructive sleep apnea (OSA) generally refers to the cessation of oral and nasal airflow for 10 seconds or more at each attack, accompanied by a decrease in blood oxygen saturation. OSA is a common respiratory disorder during sleep, presenting with repetitive apnea and hypoventilation during sleep [1]. OSA can cause hypoxemia, hypercapnia, and sleep interruption, leading to a series of pathophysiological changes. Adults often have more than 30 episodes during 7 hours of sleep every night. There are also central sleep apnea (CSA) and mixed sleep apnea (MSA). In recent years, with the continuous development of various test methods, in-depth comprehensive research on OSA has found that the disease is complex, changeable, and widespread. This disease is related to an increase in the incidence of multi-system diseases, including atrial fibrillation, heart failure, stroke, and Alzheimer's disease [2]. The incidence of OSA is about 3%–7% in adult males and about 2%–5% in adult females [3]. OSA has already become a major public health concern worldwide due to its prevalence. Therefore, OSA cannot be generally regarded as a boring sound that affects others' rest in social intercourse, but a clinical disease that needs careful examination. It can cause many serious complications.

Retinal vein occlusion (RVO) is a retinal vascular disease characterized by dilation of the retinal vein, retinal and subretinal hemorrhage, macular edema, and retinal ischemia of varying degrees. RVO is further divided into central retinal vein occlusion (CRVO) and branch retinal vein occlusion (BRVO), which is also a primary cause of blindness [4]. Currently, fundus fluorescein angiography (FFA) is the gold standard for the diagnosis of RVO [5]. The risk factors include systemic diseases such as hypertension, diabetes, arteriosclerosis, and eye diseases such as glaucoma [6]. In recent years, some reports have shown that OSA hypopnea syndrome is an independent risk factor for CRVO. The possible reason is that the patients with OSA hypopnea syndrome have not been treated for a long time, leading to hypoxia, which leads to hypertension and polycythemia, which together cause the patient's blood hypercoagulability, causing both eyes to develop at the same time. Clinicians suggest that patients should actively treat OSA hypopnea syndrome while treating CRVO [7]. Also, clinical studies have shown that OSA is related to RVO, and the mechanism below is involved: OSA causes hemodynamic changes and increases sympathetic activation, inducing oxidative stress, vascular endothelial dysfunction, increased platelet accumulation, inflammation, and metabolic disorder. These events may directly influence retinal microcirculation or work synergistically with other pathogenic factors of RVO, finally resulting in RVO [8]. Whether OSA is a risk factor for RVO remains to be confirmed by evidence-based medicine. There has been no meta-analysis investigating the correlation between OSA and RVO [9]. In this study, case-controlled studies and cohort studies involving OSA and RVO cases are collected to assess their correlation between OSA and RVO.

The remainder of this paper is organized as follows.  Section 2 discusses the related work, followed by the literature review in Section 3. The results and analysis are discussed in Section 4.  Section 5 is the meta-analysis results. Finally, we summarize the work of the full text and analyze the shortcomings of the research in Section 6.

## 2. Related Work

It is estimated that the prevalence of OSA in the general population is 3%∼7%. Obesity, family history of OSA, climacter, smoking, and alcohol consumption can increase the incidence of OSA. OSA is a group of diseases characterized by recurrent transient apnea during night sleep. In addition to the chronic impairment of systemic multiple organ function, it is often accompanied by a series of eye diseases, such as eyelid relaxation syndrome, keratoconus, and non-arteritic anterior ischemic optic neuropathy. In recent years, the correlation between OSA and eye diseases has drawn increasing attention. Previous studies have shown that OSA is a risk factor for glaucoma [10], non-arteritic anterior ischemic optic neuropathy (NAION) [11], and diabetic retinopathy (DR) [12]. The possible working mechanism is that OSA may be related to intermittent tissue hypoxia and sympathetic nerve activation stimulated by arousal, inducing oxidative stress. As a result, the abnormality occurs in the self-regulating function of ocular blood vessels, damaging the local ocular tissues and functions [13].

The characteristic chronic intermittent hypoxia of OSA may affect retinal perfusion, retinal ganglion cell (RGC) damage, and cause or aggravate eye diseases. OSA can cause changes in retinal microcirculation. Respiratory events resulting from OSA lead to hypoxia, hypercapnia, and activation of the sympathetic nervous system. Hypoxia plus sympathetic nerve activation further causes dilation of the central retinal artery with an increase in pressure. Thus, the adjacent central retinal vein is compressed. The dilation of the cerebral blood vessels resulting from hypercapnia increases intracranial pressure and cerebrospinal fluid pressure around the optic nerve head, inducing papillary edema and an increase in the venous pressure. Besides, the blood flow speed in reticular microcirculation decreases. In the meantime, persistent airway obstruction causes asphyxia. Prolonged violent fluctuation of intrathoracic pressure adversely affects the hemodynamic homeostasis of the cardiocerebral vascular system. All of the above changes are detrimental to ocular microcirculation [14]. In addition, OSA-induced intermittent hypoxia results in the generation of active oxygen species and inflammatory cytokines, which further triggers the exogenous coagulation pathway and platelet aggregation. Both active oxygen species and inflammatory cytokines can damage the repair ability of the endothelial cells [15, 16]. All of the above factors can cause a hypercoagulable state, a disorder typical of OSA, and promotes RVO. Besides, due to a higher level of retinal oxygen consumption and metabolic activity, changes secondary to OSA are more likely to affect the retina than in other positions [17].

At present, continuous positive airway pressure (CPAP) is the preferred treatment for adult OSA patients. CPAP can noticeably improve the Epworth sleepiness scale (ESS) score in OSA patients, reducing AHI and arousal index while increasing the lowest nighttime oxygen saturation [18]. It has been reported that CPAP can improve vascular reactivity, endothelial repair ability, and hypercoagulable state of patients [19, 20]. In brief, CPAP can reverse some pathological changes in RVO. However, there is still a lack of specific guiding principles and further investigation.

## 3. Materials and Methods

The present meta-analysis was conducted based on preferred reporting items for systematic reviews and meta-analyses (PRISMA) [21], which has been registered with the International Prospective Register of Systematic Reviews (No. 272373).

### 3.1. Search Strategy

Databases were searched for articles on the correlation between OSA and RVO from inception to July 14, 2021, including PubMed, Embase, Cochrane, Web of Science, CNKI, WanFang, VIP, and Chinese Biomedical Literature Database (CBM). The English search terms were as follows: sleep apnea, obstructive, obstructive sleep apnea syndrome, obstructive sleep apnea, OSA, sleep apnea syndromes, sleep hypopnea, sleep apnea, retinal vein occlusion, retinal branch vein occlusion, and central retinal vein occlusion.

### 3.2. Inclusion and Exclusion Criteria

Inclusion criteria are as follows: (1) full-text case-controlled studies or cohort studies published in any language; (2) the study population was aged ≥18 years old, regardless of race, nationality, and gender; (3) the case group recruited confirmed RVO patients (including BRVO and CRVO), and the control group recruited age- and gender-matched subjects; (4) the studies which assessed the correlation between OSA and RVO; and (5) the studies which reported the odds ratio (OR) and the 95% confidence interval (CI) or these two indicators could be calculated from the data available from the studies.

Exclusion criteria are as follows: (1) reviews or other non-primary sources; (2) non-cohort studies or cross-sectional studies; (3) studies from which valid data could not be extracted; and (4) studies involving no control populations.

### 3.3. Literature Screening and Quality Assessment

In this study, two assessors were arranged to conduct literature screening, data extraction, quality assessment, and cross check independently. The categories of information extracted from each study include: (1) project name, including the first author and the year of publication; (2) research information, including the study field, project type, and sample size; (3) baseline data, including the gender, age, and body mass index (BMI) of the subjects; and (4) diagnostic criteria, including the diagnostic criteria for RVO and OSA. During the screening, the titles and the abstracts were first read, and the studies that apparently did not conform to the inclusion criteria were excluded. The full texts of the potentially eligible studies were read. Then, it was determined whether to include the studies based on the above inclusion and exclusion criteria. In case of divergent opinions between the two assessors, a third researcher was invited for the judgment. The study quality was assessed using the Newcastle-Ottawa Scale (NOS) [22].

### 3.4. Statistical Analysis

All statistical analyses were conducted using Stata 17 software. OR and 95% CI were calculated for each study, which were used to assess the correlation between OSA and RVO. Continuous variables were described by the mean difference (MD). I2 was calculated as a measure of heterogeneity. The fixed-effects model was used if I2≤50%. The sources of heterogeneity were analyzed if I2＞50%. Besides, the use of a random-effects model was considered for the pooled analysis. Descriptive analysis or subgroup analysis was also conducted if necessary. The publication bias was assessed using the funnel plot and Egger's test. Publication bias exists if the *P*-value of Egger's test was smaller than 0.05. Otherwise, the publication bias was thought to be absent. Leave-one-out sensitivity analysis was carried out to determine the potential effect of an individual study on the overall risk assessment.

## 4. Experimental Results and Analysis

### 4.1. Search Results

Preliminary screening produced 127 studies according to the search strategy, as shown in Figure 1. After excluding the repeated ones, 75 studies were left. Then, 62 ineligible studies were excluded after reading the titles and abstracts. Among the 13 studies left, there were no control groups in 5 studies after reading the full texts; valid data could not be extracted from 2 studies. Thus, 6 studies were finally included, including 5 case-controlled studies [23–27] and 1 cohort study [28]. The total number of subjects involved in the included studies was 36,086. The cohort studies were managed based on the principles of a nested case-control study, and the results were combined with those from the case-controlled studies, as shown in Figure 1.

### 4.2. Basic Features of the Included Studies and Quality Assessment

The major characteristics of the included studies can be found in Tables 1 and 2. Six eligible studies were finally included, and they were published between 2012 and 2021. The countries included in the meta-analysis were China and France. The quality of the studies was assessed by two independent assessors using NOS, covering selectivity, comparability, and exposure factors. Data were extracted to assess each quality indicator. One point was assigned if one indicator met the criteria. A score of 9 was assigned if the included study met all of the eight indicators. If a study has scored 6 and above, this study was considered of good quality. According to the NOS assessment, the total score was ≥6 in 6 studies, including 2 studies scored 6, 2 studies scored 7, and 2 studies scored 8. In Table 1, RUSleep, FFA, and BMI represent portable monitoring device, fundus fluorescein angiography, and body mass index, respectively.

## 5. Meta-Analysis Results

### 5.1. Forest Plot of Meta-Analysis

A heterogeneity test was performed for the included studies. No significant heterogeneity was found between the studies (*p* = 0.28; I-squared = 20.3%). Thus, the fixed-effects model was used for the meta-analysis. The pooled OR was 3.24 (2.34 and 4.49), indicating that the RVO risk in OSA patients was 3.24 times the risk in the control group, as shown in Figure 2.

### 5.2. Publication Bias

The funnel plot is drawn as follows based on the OR statistic, as shown in Figure 3. It can be seen from the figure that the funnel plot is basically symmetrical. The publication bias was assessed using Egger's test, as illustrated in Table 3. *p* = 0.195 according to the results, indicating no significant publication bias. In Table 3, SE represent  standard error, OR represent odds ratio, and CI is confidence interval.

### 5.3. Sensitivity Analysis

Sensitivity analysis was conducted by excluding one study at a time from publication. The impact of an individual study on the pooled effect size was observed. It was found that excluding any study did not have a significant impact on the pooled OR value, as shown in Figure 4. The above results indicated that the present meta-analysis was robust and reliable.

## 6. Conclusions

In this study, the correlation between OSA and RVO is investigated by reviewing the case-controlled studies and cohort studies. The results confirm the correlation between OSA and RVO. Compared with the non-OSA control group, the RVO risk in OSA patients increases by over 3-fold. The pooled OR is 3.24 (95% CI, 2.34–4.49). It is clearly evident that OSA is a risk factor for RVO, which is consistent with the previous studies. It is suggested that OSA patients, especially those combined with vasculopathy such as hypertension should receive ophthalmoscopy and FFA screening to facilitate an early diagnosis and treatment of RVO. The study also has some limitations: first, the sample size is small, and the results of the meta-analysis remain to be further verified through more prospective studies. Second, due to the small sample size, we do not analyze the confounding factors or assess the influence of OSA on different types of RVO. Third, the population included in the meta-analysis came from a limited number of regions, and the research results need to be verified by more ethnic or regional populations. In future, more high-quality prospective studies should be conducted to verify the correlation between OSA and RVO.

## Figures and Tables

**Figure 1:** Flow diagram of study selection.

**Figure 2:** Forest plots showing risk estimates of the association.

**Figure 3:** Begg's funnel plot.

**Figure 4:** Sensitivity analysis of the included studies.

**Table 1:** Characteristics of included studies.

Study	Study Design	TotalNumber	Nation	Case group				Control group				OSA Diagnostic methods	RVO Diagnostic methods
				Male(%)	Age (years)	BMI	Number	Male (%)	Age (years)	BMI	Number		
Wan et al. 2021 [23]	Case-control study	90	China	17 (38)	60.07 ± 10.33	28.18 ± 6.25	45	25 (56)	60.33 ± 9.46	24.80 ± 6.04	45	PSG	FFA
Leung and Wang 2020 [24]	Case-control study	140	China	45 (64)	59.75 ± 13.69	25.12 ± 5.39	70	45 (64)	57.16 ± 12.95	24.37 ± 3.89	70	PSG	FFA
Wang et al. 2019 [25]	Case-control study	60	China	18 (60)	52.51 ± 11.72	26.87 ± 4.45	30	19 (63)	50.79 ± 12.43	24.64 ± 3.46	30	PSG	FFA
Chen et al. 2019 [26]	Case-control study	48	China	17 (71)	50.71 ± 9.49	25.49 ± 4.17	24	17 (71)	51.07 ± 8.97	22.57 ± 5.25	24	PSG	FFA
Agard et al. 2018 [27]	Case-control study	114	France	30 (43)	71.6 ± 11.7	26.70 ± 4.60	69	20 (44)	73.80 ± 6.70	25.70 ± 3.80	45	RUSleep	FFA
Chou et al. 2012 [28]	Cohort study	35634	China	―	―	―	52	―	―	―	35582	―	―

**Table 2:** Assessment of study quality.

Inclusion study	Selection	Comparability	Exposure	Total
Wan et al. 2021 [23]	4	2	2	8
Li et al. 2020 [24]	3	2	2	7
Wang et al. 2019 [25]	3	2	2	7
Chen et al. 2019 [26]	4	2	2	8
Agard et al. 2018 [27]	3	1	2	6
Chou et al. 2012 [28]	3	1	2	6

**Table 3:** Egger's test published bias test results.

Std_Eff	Coef.	SE.	t	*p* > |*t*|	[95% CI]	
Slope	−0.0177	0.771336	−0.02	0.983	−2.15927	2.123872
Bias	2.826938	1.819166	1.55	0.195	−2.22388	7.877753

## Data Availability

The simulation experiment data used to support the findings of this study are available from the corresponding author upon request.
